The article "Infraocclusion: Prevalence, Characteristics, and Associated Dental Anomalies in Arabian Children" was published in 2022. Journal: Biomed Res Int.

# Infraocclusion: Prevalence, Characteristics, and Associated Dental Anomalies in Arabian Children

**DOI:** 10.1155/2022/6624804

**Published:** 2022-07-23

**Authors:** Saleh Ibrahim Alshaya, Abdulrahman Faleh Alanazi, Saleh Sulaiman Aldawish, Mogren Mohmed Alsuhaim, Mohammad Saad Alomar, Yazeed Marzouq Almuaytiq, Sami Abdulaziz Alfahad, Abdulrahman Abdulmohsen Suliman Almousa, Abdullah Alassaf, Sreekanth Kumar Mallineni

**Affiliations:** ^1^College of Dentistry, Majmaah University, Al-Majmaah 11952, Saudi Arabia; ^2^Department of Preventive Dental Science, College of Dentistry, Majmaah University, Al-Majmaah 11952, Saudi Arabia; ^3^Center for Transdisciplinary Research (CFTR), Saveetha Institute of Medical and Technical Sciences, Saveetha Dental College, Saveetha University, Chennai, 600077 Tamil Nadu, India; ^4^Division for Globalization Initiative, Liaison Center for Innovative Dentistry Graduate School of Dentistry, Tohoku University, Sendai, Japan

## Abstract

**Aim:**

To analyze the distribution and characteristics of infraocclusion among Arabian children in primary dentition and its associated dental anomalies.

**Methods:**

A radiographic analysis was performed retrospectively using digital panoramic radiographs of children attending the pediatric dental clinic of College of Dentistry, Majmaah University, Saudi Arabia, from January 2019 to May 2021. The panoramic radiographs were analyzed to assess the distribution and characteristics of infraocclusion and its associated dental anomalies. Descriptive statistics were used for comparisons using SPSS version 21.0 (IBM Corp., Armonk, N.Y., USA). The chi-square test was used to compare percentages.

**Results:**

Among the study population (542), only 40 children reported infraocclusion of 65 primary molars. Infraocclusion was common in males (90%) and very frequent in the mandibular arch (*n* = 48 teeth). In the primary dentition, unilateral infraocclusion (62.5%) was very frequent than bilateral presence (37.5%). Single molars were involved in 50% of the patients, while two, three, and four molars were involved in 42.5%, 2.5%, and 5% of cases. The mandibular second primary molar was frequently affected with infraocclusion, while the maxillary first primary molar was less commonly affected. In the mandibular arch, the second primary molar (28, 58%) was more commonly affected with infraocclusion than the mandibular first primary molars and maxillary primary and secondary molars (*p* < 0.05). The majority of the infraoccluded molars were mild (75%), followed by moderate (23.5%) and severe (1.5%). Hypodontia (12.5%) is frequently associated with infraocclusion, followed by supernumerary teeth (5%) and radix entomolaris of the first permanent mandibular molars (5%). Infraocclusion was more in the second primary molar mandibular arch, while in the maxillary arch, the first primary molars were commonly affected (*p* > 0.05).

The article "Infraocclusion: Prevalence, Characteristics, and Associated Dental Anomalies in Arabian Children" was published in 2022. Journal: Biomed Res Int.

**Conclusion:**

In Arabian children, infraocclusion was commonly observed in mandibular second primary molars. Unilateral infraocclusion is a mild type of infraocclusion frequent in Arabian children. Numerical anomalies such as hypodontia and supernumerary teeth are associated with infraocclusion.

## 1. Introduction

Infraocclusion is a clinical finding in which teeth are found below the occlusal surface compared to adjacent teeth. Numerous terms have been used, like half retention, arrested eruption, buried tooth, tooth depression, retained deciduous tooth, shortened tooth, disillusion, impaction, incomplete/suppressed eruption, intrusion, secondary retention, and reinclusion. Nonetheless, the most frequently used terms are infraocclusion, ankylosed tooth, and submerged tooth [1], which refer to the chief visual feature of the abnormality. They have become the term of preference for this positional anomaly of teeth [2, 3]. In most cases, infraocclusion can be appreciated clinically, but radiographic examination is seldom required to diagnose this entity [1, 4]. This developmental dental anomaly may occur if the tooth eruption mechanism fails and subsequently alters the preservation of its vertical position to the neighboring tooth [5–9]. Typically, the marginal ridges of the infraoccluded tooth are below the adjacent teeth. Ankylosis is a common reason for infraocclusion. It happens because of the failure of the periodontal ligament to separate the root from the alveolar bone, which results in the fusion of the bone and root [6–8]. The classification of infraocclusion has been discussed by various authors; however, the Brearley classification has been used by various researchers in literature [10]. The classification involves three types that include (i) mild (occlusal surface located approximately 1 mm below the occlusal plane of the adjacent tooth), (ii) moderate (occlusal surface at the level of the contact point to the adjacent tooth), and severe (occlusal surface level below the interproximal gingival tissue of adjacent tooth). The reported prevalence of infraocclusion varies broadly. An American study [11] reported a prevalence of 1.3% in 2342 schoolchildren, a study from Israel [10] reported 24.8% among 1530 children, and a Swedish study [1] reported 8.9% in 1059 children. Infraocclusion is very common in primary dentition rather than permanent dentition. It is primarily seen in the mandibular arch as compared to the maxillary arch. Infraocclusion in primary molars has been linked with a few other dental anomalies. These include an ectopic eruption of the first permanent molars, peg-shaped lateral incisors, palatal displacement of maxillary canines, and enamel hypoplasia [12, 13]. Another aspect thought to play a role in infraocclusion is hypodontia. In a study, 65.7% of patients with missing permanent premolars reported having infraoccluded primary molars [14, 15]. The high occurrence of infraocclusion in patients with hypodontia recommends a possible common aetiological mechanism [16, 17]. The novelty of the present study is the lack of studies on the prevalence of infraocclusion in primary dentition and its associated anomalies among Arabian children. Hence, the present study was aimed at analyzing the distribution and characteristics of infraocclusion among Arabian children in primary dentition and its associated dental anomalies.

The article "Infraocclusion: Prevalence, Characteristics, and Associated Dental Anomalies in Arabian Children" was published in 2022. Journal: Biomed Res Int.

## 2. Materials and Methodology

A retrospective cross-sectional radiographic analysis was performed using digital panoramic radiographs of children attending the pediatric dental clinic of College of Dentistry, Majmaah University, Saudi Arabia, from January 2019 to May 2021. The institutional ethical committee of Majmaah University, Saudi Arabia, approved the study.

### 2.1. Inclusion Criteria

Healthy children with clear panoramic radiographs of Arabian origin were included. Radiographs of children aged 4 to 12 years and those with eight primary molars were considered for further analysis.

### 2.2. Exclusion Criteria

The children with blurred or poor-quality radiographs, children other than the Arabian origin, and children with systemic problems or growth retardation, cleft lip and palate, and other syndromes were excluded. Children more than 12 years of age and less than four years of age and with absence of any primary molars, incomplete records, and parental informed consent were not considered.

### 2.3. Procedure

The 542 panoramic radiographs were analyzed to assess the distribution and characteristics of infraocclusion and its associated dental anomalies. The data collection included is based on the gender of the child (male and female), age, the number of molars affected (1, 2, 3, 4, 5, 6, 7, and 8), arch (maxillary and mandibular), and type of infraocclusion [10] (Figure 1) (mild, moderate, and severe). Associated dental anomalies like tooth agenesis/hypodontia, a supernumerary tooth, odontomas, tooth transposition, impacted teeth, and other dental anomalies were also evaluated.

### 2.4. Statistical Analysis

All data tabulated and descriptive statistics were used for comparisons using SPSS version 21.0 (IBM Corp., Armonk, N.Y., USA). The chi-square test was used to compare percentages, and a *p* value was considered less than 0.05. Kappa statistics were used to identify intra- and interexaminer reliability.

The article "Infraocclusion: Prevalence, Characteristics, and Associated Dental Anomalies in Arabian Children" was published in 2022. Journal: Biomed Res Int.

## 3. Results

Among the radiographs of 542 children included in the study, only 40 (7.38%) children reported infraocclusion of 65 primary molars. The infraocclusion was primarily seen in 36 (90%) males as compared to 4 (10%) females. Unilateral infraocclusion (62.5%) was very often compared to bilateral presence (37.5%) in the primary dentition (Table 1). Single molars were involved in 50% (20) of the children, while two, three, and four molars were involved in 42.5% (17), 2.5% (1), and 5% (2) of the cases (Figure 2). In the mandibular arch, the second primary molar (28, 58%) was commonly affected with infraocclusion, followed by the first primary molar (20, 42%), while in the maxillary arch, the first primary molars (9, 53%) were more frequently affected than the maxillary second primary molar (8, 47%); the findings were statistically significant (*p* < 0.05). Among infraoccluded primary molars, 55% were primary second molars and 45% were first primary molars. Among the infraoccluded molars, right second primary molars and maxillary right first primary molars were commonly affected. The majority (75%) of the infraoccluded molars were mild in nature followed by moderate (23.5%), and 1.5% (1) were the severe type of malocclusion (Figure 2); the comparison was not statistically significant (*p* > 0.05). Hypodontia (12.5%) was frequently associated with infraocclusion, followed by supernumerary teeth (5%) and radix entomolaris of the first permanent mandibular molars (5%) (Figure 3). The findings were not statistically significant (*p* > 0.05). Kappa statistics confirmed substantial interrater reliability between the two examiners (kappa = 0.86).

## 4. Discussion

Infraocclusion of the deciduous molar is a common finding in which the tooth fails to reach the occlusal level compared to the adjacent teeth. Though infraocclusion can be clinically diagnosed, in children, assessing its severity is tough, so dental radiographs are a boon in assessing such anomalies. Panoramic or intraoral periapical radiographs and computed tomography (CT) can determine the space between the infraoccluded tooth surface and the normally occluded adjacent teeth [18]. The present study was conducted to assess the prevalence of infraocclusion in Arabian children using panoramic radiographs attending a teaching hospital. This retrospective analysis was done to determine the incidence and importance of infraocclusion of primary molars and to report other associated dental anomalies in Arabian children using panoramic radiographs, even though the etiology of infraoccluded teeth remains unclear. The following factors can be considered: disturbing local metabolism, periodontal membrane disorders, trauma or infection, thermal or chemical irritation, systemic diseases (like congenital syphilis), hereditary cause, local failure of bone growth, unusual pressure from the tongue, disturbance in the typical hard tissue resorption and deposition, and lack of space [4, 18, 19].

The article "Infraocclusion: Prevalence, Characteristics, and Associated Dental Anomalies in Arabian Children" was published in 2022. Journal: Biomed Res Int.

Infraocclusion might be age-dependent, as it is closely associated with root resorption due to premolar eruption and the process of normal shedding. Peretz et al. [5] reported that there was a rise in the moderate form (8-10 years old) and severe form (11-13 years) [5]. In a study by Sidhu and Ali, the severe infraocclusion affected around 2.5–8.3% of the total infraoccluded primary molars [20]. In line with previous findings, the present study included subjects ranging from 2 years and inferred that infraocclusion occurred at a mean age of 9.2 ± 3.8 years. The reported prevalence of infraocclusion among children varies from 2.8% to 38.5% according to various studies [1, 2, 16, 21–27] published in the literature (Table 2).

Kurol [13] through clinical observation of 1059 children between 3 and 12 years of age observed that females between 3 and 6 years old showed more infraoccluded teeth, whereas male children suffered from this condition more between 7 and 12 years of age [13]. The incidence of infraocclusion of deciduous second molars is more or less the same between males and females, as described by Silvestrini Biavati et al. [21]. According to the findings reported by previous studies, there was an insignificant difference in the prevalence of infraocclusion with regard to gender, according to the findings reported by previous studies [10, 16, 28]. On the contrary, Steigman et al. described a higher incidence of ankylosed mandibular second molars in males [22]. Ciftci et al. [23] reported that there was no statistically significant difference in the prevalence of infraocclusion between girls (*n* = 51) and boys (*n* = 73). However, the present study noticed more incidence in males compared to females. The occurrence of infraocclusion of primary molars is reported to be in the 1.3-8.9% [1]; however, it can be as high as 38.5% [28]. Silvestrini Biavati et al. collected a group of 512 Italian subjects aged between 5 and 15 years and found an incidence of ankylosis of 6.6% [21]. Furthermore, the results of the present study revealed that the occurrence of infraocclusion is more frequent in second primary molars; this anomaly has higher percentages in the mandibular arch than in the maxillary arch. In children with such developmental abnormalities, space issues might pose and in such cases expansion may become essential [18, 29, 30]. According to previous studies, the prevalence of mandibular infraocclusion was more than that of maxillary infraocclusion (189 : 36), and in the mandibular arch, the incidence is 2 to 10 times higher than that of the maxillary arch [1, 2, 21–24]. Overall, infraocclusion affects predominantly mandibular molars up to 27 times more according to Odeh et al. [16]. In a study by Venza et al., subjects exhibited multiple infraoccluded teeth; the total number of infraoccluded teeth was 225, with a mean value of 1.7 infraocclusion per child [2]. Also, Zuñiga et al. [24] and Salem and Mirzaee [25] reported 1.9 and 2.1 infraocclusions per child, respectively. However, Brearley and McKibben [10] and Kurol [1] reported higher percentages of infraocclusion affecting only one molar per child (51% and 52%, respectively). This data is consistent with similar results of the present study, which showed that around 50% of subjects had multiple infraoccluded teeth.

The article "Infraocclusion: Prevalence, Characteristics, and Associated Dental Anomalies in Arabian Children" was published in 2022. Journal: Biomed Res Int.

A Turkish study [23] examined 3.5% of the study population, and the authors reported that 45.2% involved one tooth, 47.6% involved two teeth, 3.2% involved three teeth, and 4% involved four or more teeth with infraocclusion. In the present study, half of the children with infraocclusion involved a single tooth; 42.5% involved two infraoccluded molars, while 3 and 4 infraoccluded molars were 2.5% and 5%, respectively. The present study included children with eight primary molars, and Turkish was mentioned regarding the presence of primary molars. According to Bjerklin and Bennett's method, the most observed category of infraocclusions was the mild one [31]. The results of the present study are consistent with the report of Brearley and McKibben [10] and Cardoso Silva et al. [26] and Venza et al. [2]. They used the same method, with infraoccluded molars mild in nature (75%) followed by moderate (23.5%) and severe (1.5%). Silvestrini Biavati et al. also described similar findings using different classifications [21]. In the presence of infraoccluded primary molars, successor permanent teeth may also get affected, and a delay in development can occur in those teeth. In a study by Ciftci et al. [23], dental variation was seen in 50.8% of children with infraocclusion. The dental anomalies accompanying infraocclusion were mostly agenesis, followed by dens invaginatus and supernumerary tooth. Shalish et al. [3] reported an increased rate of dental anomalies associated with infraocclusion of primary molars, palatally displaced canines, tooth agenesis, microdontia of maxillary lateral incisors, and distal angulation of the mandibular second premolars [3]. Other associated anomalies reported are aplasia of a successor, supernumerary teeth, radix entomolaris of permanent teeth, and high prevalence of agenesis [16, 25, 26]. Most of the authors observed that the primary molars without successors have more chances of infraocclusion [22, 24]. The present study reported that hypoplasia is the most common associated anomaly, followed by supernumerary teeth and radix entomolaris of permanent teeth. Further, in a study by Venza et al., significant association was observed between the occurrence of infraocclusion and impacted teeth (*p* < 0.001) [2]. However, there was no significant relation evident in the association between infraocclusion and dental anomalies in the present study (*p* > 0.05). Prior studies report an association with multiple anomalies [32–39] with infraocclusions. The concomitant occurrence of various development anomalies may be coincidental; however, the exact etiopathology was not clearly understood [40]. On the contrary, Lochib et al. [41] find the presence of dental anomalies in 1000 schoolchildren of 3–5 years old in Faridabad. Infraocclusion (submerged teeth) concerning the deciduous molar was not observed in any of the cases. The children with infraoccluded teeth must be regularly followed up for infraocclusion at other sites [13, 42, 43]. It was suggested that the number of infraoccluded teeth could influence the decision to extract the teeth or observe the patient. Having numerous infraoccluded teeth can increase space loss or play a part in patient management if multiple extractions are required [42–44].

The article "Infraocclusion: Prevalence, Characteristics, and Associated Dental Anomalies in Arabian Children" was published in 2022. Journal: Biomed Res Int.

### 4.1. Strengths and Limitations

The first limitation of the study could be its retrospective nature and lack of quantitative measurements. Another limitation is a long-term evaluation or follow-up of patients with infraocclusion. Studies should be conducted to evaluate the changes in the severity of infraocclusion with age, including study samples with a wider age range. To the authors' best knowledge, this study is one of the recent studies, and very few studies involved subjects with all primary molars.

## 5. Conclusion

From the present study results, it can be concluded that infraocclusion was prevalent only in 7.38% of children. It was commonly observed in mandibular second primary molars. Unilateral occurrence of mild type of infraocclusion was very frequent in Arabian children. Numerical anomalies such as hypodontia and supernumerary teeth are associated with infraocclusion. Patients with such clinical findings must be regularly followed up to assess the severity, and further management must be done accordingly.

The article "Infraocclusion: Prevalence, Characteristics, and Associated Dental Anomalies in Arabian Children" was published in 2022. Journal: Biomed Res Int.

## Figures and Tables

**Figure 1:** Reference used for diagnosis of infraocclusion.

**Figure 2:** Distribution of 65 infraoccluded primary molars based on gender (a), arch (b), number of teeth (c), and type of infraocclusion (d).

**Figure 3:** Dental anomalies associated with infraocclusion.

**Table 1:** Distribution of infraocclusion among Arabian children.

Variables	*N*	%
Mean age (years)	Mean 9.2	SD 3.8
Gender		
Male	36	90
Female	4	10
Occurrence		
Unilateral	25	62.5
Bilateral	15	37.5

**Table 2:** Reported prevalence of infraocclusion.

Author	Country	Year	Incidence/prevalence	Most common tooth
Venza et al. [2]	Italy	2018	2.8%	Mandibular second primary molars
Ciftci et al. [23]	Turkey	2021	3.25%	Mandibular second primary molar
Brearley and McKibben [27]	United States of America	1973	6.9%	Mandibular first primary molar
Kurol et al. [1]	Sweden	1984	8.9%	Not mentioned
Silvestrini Biavati et al.	Italy	2011	6.6%	Mandibular second primary molars
Zúñiga-Tertre et al.	Spain	2004	10.48%	Mandibular first primary molar
Salem and Mirzaee [25]	Iran	2009	15%	Mandibular first primary molar
Cardoso Silva [26]	Spain	2014	21.8%	Mandibular first primary molar
Odeh et al. [16]	Finland	2016	Maxilla: <1%; mandible: 22%	Mandibular first primary molars
Steigman et al. [22]	Israel	1973	38.5%	First primary molars
Present study	Saudi Arabia	2022	7.3%	Mandibular second primary molars

## Data Availability

The raw data supporting the conclusions of this article will be made available by the authors without undue reservation.
